# Relationship between Artificial Intelligence-Based General Anesthetics and Postoperative Cognitive Dysfunction

This article has been retracted.

**DOI:** 10.1155/2021/5553029

**Published:** 2021-04-01

**Authors:** Xiaokun Wang, Shan Huang

**Affiliations:** ^1^Department of Anesthesiology, Tianjin Medical University Cancer Institute and Hospital, National Clinical Research Center of Cancer, Tianjin 300060, China; ^2^Key Laboratory of Cancer Prevention and Therapy, Tianjin 300060, China; ^3^Tianjin's Clinical Research Center for Cancer, Tianjin 300060, China; ^4^Nankai University, Tianjin 300071, China

## Abstract

Postoperative cognitive dysfunction (POCD) refers to the complications of the central nervous system before and after surgery in patients without mental disorders. Many studies have shown that surgical anesthesia may cause POCD, especially in elderly patients. This article aims to study the relationship between artificial intelligence-based general anesthetics and postoperative cognitive dysfunction. This article first describes and classifies artificial intelligence, introduces its realization method, machine learning algorithms, and briefly introduces the basic principles of regression and classification methods in machine learning; then, the principles and techniques of general anesthetics are proposed. The pathogenesis of postoperative cognitive dysfunction (POCD) is explained in detail. Finally, the effect of anesthetics on postoperative cognitive dysfunction is obtained from both inhaled anesthetics and intravenous anesthetics. The impact on postoperative cognitive function is explained. The experimental results in this article show that there is no statistically significant difference in the two groups of patients' age, gender ratio, body mass index, education level, preoperative comorbidities, and other general indicators. Through the use of EEG bispectral index monitors to monitor the depth of anesthesia and postoperative cognitive dysfunction, first, there was no obvious relationship between the occurrence of postoperative cognitive dysfunction at 1, 5, 10, and 50 days and discharge time. The comprehensive monitoring group can reduce the clinical dose of preventive medication and cis-atracurium and shorten the patient's recovery time, extubation time, and recovery time. In addition, it can also reduce the increase of serum protein S100*β* in elderly patients and reduce the incidence of early postoperative cognitive dysfunction.

## 1. Introduction

With the advent of an aging society and the development of medical technology [1], the types and numbers of interventions in the elderly have increased, there have been more and more studies on interventions in the elderly, and occupational diseases and complications of the elderly have become more and more serious. POCD is a complication of the central nervous system, which has a great impact on the elderly after surgery. Most of these are temporary, but there are also long-term cognitive impairments and persistent cognitive impairments. POCD not only affects the quality of life of the elderly but also brings about a greater burden to the family and society.

When the complication of postoperative cognitive dysfunction occurs, the patient may have a worse prognosis of the disease or a longer time, and it may also cause the patient's hospital stay to be prolonged and new complications to appear, therefore, people with dysfunction face high medical expenses and low prognostic quality of life. However, the current research points out that there are no exact drugs or technical methods for the treatment of postoperative cognitive dysfunction. With the attention and exploration of scholars, the risk factors and pathogenesis of cognitive dysfunction have found a new direction for the treatment of postoperative cognitive dysfunction.

Fuminori conducted research on the use of artificial intelligence (AI) in patent search in the chemical field [2], especially the efficiency research on patent search using sentences as training data. He reported on the impact of feature declarations in the field of chemistry on invalid searches and the impact of training sentences on existing technology searches. As a further AI application, he will report the investigation results of the classification of patent documents of unknown patent classification based on the results of patent documents of known patent classification. However, artificial intelligence is still in the development stage, and the realization process will be more complicated [3]. Postoperative cognitive dysfunction is a phenomenon related to increased postoperative morbidity, mortality, and resource utilization. Umholtz and Nader reviewed many studies to better characterize the biochemical basis of related cognitive dysfunction, with particular attention to the interaction between the cholinergic system and innate immunity and how the regulation of the immune system promotes related neuroinflammation. Although postoperative cognitive dysfunction has a clinical impact, there is still a lack of evidence-based prevention and treatment of these diseases. Some previous trials attempted to prevent or treat clinical manifestations by modulating the cholinergic system with acetylcholinesterase inhibitors, but the results were largely ambiguous at best [4]. The search for drugs that induce faster induction and faster recovery in the operating room has produced many anesthetics. The mechanism of action and potential side effects are still unknown, especially in young and aging brains. Armstrong et al. use their expertise in clinical and basic science to give readers an interesting view on the current applications of general anesthetics and provide evidence that they have neurotoxic effects on the developing brain and the brain of the elderly. Although the evidence collected from animal studies shows that general anesthesia can cause neurodegeneration and cognitive impairment, so far, a clear consensus on the effects of anesthetics on humans is still elusive [5].

The innovation of this article is summarized as follows: (1) It provides an analysis of the impact of different anesthesia management methods on the occurrence of early and long-term cognitive dysfunction in elderly patients after surgery. (2) Combined with sodium creatine, it is confirmed that it has obvious effect on the treatment of left heart failure in the elderly, and it is worthy of clinical application to help patients recover quickly. (3) The use of two-way EEG indicators to monitor the depth of anesthesia can effectively reduce the incidence of postoperative cognitive impairment.

## 2. Application of Artificial Intelligence Algorithms in the Relationship between General Anesthetics and Postoperative Cognitive Dysfunction

### 2.1. Artificial Intelligence Algorithm

By observing the development history of artificial intelligence technology, the realization of artificial intelligence can be divided into five types of groups: symbolism, connectivity, learning, action, and evolution [6]. There is no difference between these 6 methods, but solutions are proposed from various angles. For example, in learning and education, artificial neural networks are used for success. The current popular machine learning and deep learning algorithms are actually symbolic and connected and action further expanded [7–9].

To understand mechanical learning, you can start with three questions, namely, what to learn, how to learn, and what to do [10, 11]. At present, behind more artificial intelligence applications is the process of removing real problems in the corresponding mathematical models [12]. They are broken down into the organic combination of these three core works and their modeling and resolution.

Society is constantly advancing, science is developing rapidly, machine learning technology is also greatly improved, and methods for regression and classification are also increasing, such as LS (least squares), PLS (partial least squares), SVM (support vector machine), and GP (Gaussian process). The basic principles of these common methods are usually well known [13, 14].

#### 2.1.1. Principles and Characteristics of LS

Least-squares method is an optimization technique. The main idea is to minimize the sum of squared errors between different data, so as to find the best match of the data function [15]. Unknown data can be easily obtained through the block method, and the sum of squares of the difference between the requested data and the actual data is the smallest. The least-squares method can also be used to place curves [16]. The basic principles are as follows.

If there is a univariate linear normal error model relationship between *y* and *x* in the population, then, for given *x*_*i*_, there are

(1) $$\begin{array}{c} y_{i}=B_{0}+B_{1}x_{i}+\xi_{i}. \end{array}$$

Let the estimated parameter be ${\hat{B}}_{0}=b_{0},{\hat{B}}_{1}=b_{1}$. Assuming that a certain method is used to find the estimated values *b*_0_ and *b*_1_, the estimated equation can be obtained:

(2) $$\begin{array}{c} {\hat{y}}_{i}=b_{0}+b_{1}x_{i},\;i=1,2,\ldots ,n. \end{array}$$

For each *x*_*i*_, this estimation equation has a certain ${\hat{y}}_{i}$ corresponding to it. Obviously, its value is often not equal to the actual observation value, but there is a deviation *c*_*i*_; namely,

(3) $$\begin{array}{c} c_{i}=\left(y_{i}-{\hat{y}}_{i}\right). \end{array}$$

*c*_*i*_ is sometimes called residual. In order to express the deviation of all observed values from the regression estimates, the sum of squared residuals is generally considered:

(4) $$\begin{array}{c} \overset{n}{\underset{i=1}{\sum }}c_{i}^{2}=\sum_{i=1}^{n}{\left(y_{i}-{\hat{y}}_{i}\right)}^{2}=\overset{n}{\underset{i=1}{\sum }}{\left(y_{i}-b_{0}-b_{1}x_{i}\right)}^{2}. \end{array}$$

In a geometric sense, a good regression equation should be able to minimize the sum of squares of estimated deviations. Therefore, the problem comes down to finding the estimated parameters *b*_0_ and *b*_1_ so that the following formula is satisfied:

(5) $$\begin{array}{c} \overset{n}{\underset{i=1}{\sum }}c_{i}^{2}=\overset{n}{\underset{i=1}{\sum }}{\left(y_{i}-b_{0}-b_{1}x_{i}\right)}^{2}⟶\min. \end{array}$$

Using the method of obtaining partial derivatives, *b*_0_ and *b*_1_ can be obtained. Obviously, when the variables *x* and *y* are standardized variables, the regression equation is

(6) $$\begin{array}{c} \hat{y}=u_{xy}x. \end{array}$$

Among them, *b*_1_=*u*_*xy*_.

The above is a one-variable linear regression. For multivariable linear regression, *y* is still recorded as the dependent variable. When there are *q* independent variables *x*_1_, *x*_2_,…, *x*_*q*_, the theoretical model is

(7) $$\begin{array}{c} y=B_{0}+B_{1}x_{1}+\cdots +B_{q}x_{q}+\xi . \end{array}$$

Write this model in matrix form, and remember that

(8) $$\begin{array}{c} Y={\left[\begin{array}{c} y_{1}\\ y_{2}\\ \vdots \\ y_{n} \end{array}\right]}_{n\times 1},\\ X={\left[\begin{array}{ccc} 1 & x_{11} & x_{1q}\\ 1 & x_{21} & x_{2q}\\ \vdots & \vdots & \vdots \\ 1 & x_{n1} & x_{nq} \end{array}\right]}_{n\times \left(p+1\right)},\\ B={\left[\begin{array}{c} B_{0}\\ B_{1}\\ \vdots \\ B_{q} \end{array}\right]}_{\left(p+1\right)\times 1},\\ \xi ={\left[\begin{array}{c} \xi_{1}\\ \xi_{2}\\ \vdots \\ \xi_{n} \end{array}\right]}_{n\times 1}. \end{array}$$

The matrix multivariable linear regression model is

(9) $$\begin{array}{c} Y_{n\times 1}=X_{n\times \left(p+1\right)}B_{\left(p+1\right)}+\xi_{\left(n\times 1\right)}. \end{array}$$

Through the calculation method of least squares, the normal equation can be obtained:

(10) $$\begin{array}{c} X^{T}XB=X^{T}Y. \end{array}$$

Since *x*_1_, *x*_2_,…, *x*_*q*_ does not have a complete correlation assumption (i.e., the rank of *X* is *p*), *X*^*T*^*X* is an invertible matrix [17]. Therefore, the least-squares estimator of the overall parameter is obtained:

(11) $$\begin{array}{c} D_{\text{LS}}={\left(X^{T}X\right)}^{-1}X^{T}Y. \end{array}$$

The least-squares estimator of *Y* is

(12) $$\begin{array}{c} \hat{Y}=X{\left(X^{T}X\right)}^{-1}X^{T}Y. \end{array}$$

LS is a linear regression method. The method is simple and easy to implement. It is unbiased. In the actual industrial process, a large sample size is required [18, 19].

#### 2.1.2. The Basic Principle of SVM

Support vector machine is abbreviated as SVM. When used for classification problems, for a given set of samples, the training set is as follows:

(13) $$\begin{array}{c} \left(x_{1},y_{1}\right),\left(x_{2},y_{2}\right),\ldots ,\left(x_{M},y_{M}\right),\;x\in R^{d},y\in R, \end{array}$$

where *d* is the dimension of the actual input data space. The decision function of SVM is based on the symbols of the following formula:

(14) $$\begin{array}{c} f\left(x\right)=\sum_{i=1}^{M}y_{i}a_{i}H_{h}\left(x_{i},x\right)+b. \end{array}$$

In the formula, *M* represents the number of samples, AAA is the kernel function mapping the input vector to the feature space, *h* represents the set of several parameters, and *b* represents the deviation [20, 21]. The coefficient *a*_*i*_ in the formula is obtained by solving the following quadratic optimization problem:

(15) $$\begin{array}{c} w\left(a\right)=\sum_{i=1}^{M}a_{i}-\frac{1}{2}\sum_{i=1}^{M}\sum_{i=1}^{M}a_{i}a_{j}y_{i}y_{j}H_{h}\left(x_{i},x_{j}\right). \end{array}$$

There is 0 ≤ *a*, *i*=1,2,…, *M*, which is the following constraint:

(16) $$\begin{array}{c} \sum_{i=1}^{M}a_{i}y_{i}=0. \end{array}$$

Since the above optimization problem does not consider the training error, it is called a hard limit optimization problem. The specific transformation of the core function is as follows:

(17) $$\begin{array}{c} H\leftarrow H+\frac{1}{C}. \end{array}$$

### 2.2. Principles of General Anesthetics

General anesthesia undoubtedly acts on the central nervous system, including the brain and spinal cord. It can temporarily eliminate the reflexes of the consciousness and sensory nervous system and relax the skeletal muscles. It is mainly used for surgical anesthesia. General anesthesia acts on the central nervous system and affects the release of buttons and the connection of receptors: general anesthesia plays an important role in the activation of GABA and midazolam glycine receptors in the central nervous system and may prolong hippocampal neuronal activity [22]. It has an obstructive effect on the central choline working system and the N-methyl-D-asparagine (NMDA) receptor function; it can regulate the neuronicotine receptor, serotonin working receptor, and adrenaline working receptor. Function is the basis for general anesthetics to exert the molecular mechanism of anesthesia. These results mainly affect ion channels in cell membranes and hinder the transmission of information, resulting in anesthetic effects. GABA receptors in the hippocampus play an important role in learning and memory and have an important impact on cognitive functions [23].

### 2.3. Pathogenesis of POCD

The pathogenesis of POCD before El is unclear. It is generally believed that POCD is based on central nervous system degeneration, which is caused or exacerbated by various stress stimuli [24]. The anxiety factors leading to neurodegeneration include physical factors (surgery), chemical factors (anesthesia and drugs), biological factors (nutrition), and social factors (mental stress), including central nervous system disorders, endocrine, and the three main nerves of oxidative stress [25, 26]. The possible mechanisms are the following:

1. Immune system disorder
2. Surgery may cause inflammation and cause systemic acute phase reactions, which may lead to a variety of behaviors and cause psychological changes, such as loss of appetite, decreased social activities, fever, and hyperalgesia [27]. The inflammatory response may cause the peripheral and central nervous system to be more sensitive to interferon-6, and interleukin-1 and tumor necrosis factor-a affect cognitive function.
3. Oxidative stress
4. Oxidative stress and oxidative damage have been the research hotspots in recent years. The ischemic process caused by surgery, the hypoxia caused by anesthesia, and the inflammatory response can all cause oxidative damage, which will produce a large amount of reactive oxygen species and cause damage to nerve cells [28, 29]. Studies have shown that the amount of formaldehyde in the urine of patients with cognitive impairment is increasing.
5. Neuroendocrine disorders
6. The increase of age leads to the decline of endocrine function, so it is difficult to make up for the endocrine disorders caused by surgery. Neuroendocrine disorder is an important mechanism leading to cognitive impairment [30]. According to research, hypothyroidism may cause severe cognitive impairment. Evidence that is closely related to the release of thyroid pumps shows that nerve growth factors are closely related to the function of the hippocampus and play an important role in the process of neurodevelopment and learning and memory. Other studies have shown that neuroendocrine disorders may affect the appearance of L-2. This also means that it is closely related to the occurrence of cognitive impairment [31].

### 2.4. Influence of Anesthetics on Postoperative Cognitive Dysfunction

#### 2.4.1. Inhaled Anesthetics

POCD in the elderly may be related to decreased levels of acetylcholine in the brain, cholinergic neurodegeneration, and decreased number of cholinergic receptors. Inhaled anesthetics have complex and diverse effects on learning and memory functions and may significantly hinder the intake of choline by nerve cells, reducing the speed of acetylcholine synthesis. Many studies have shown that general anesthetics, such as inhaled doses below the anesthetic amount of general anesthetics, may hinder the function of the receptor. Isoflavones can activate GABA receptor activity, block NMDA receptors, reduce the release of acetylcholine, and have a great impact on cognitive functions such as learning and memory [32]. Animal experiments have shown that isoflurane can promote the appearance of Cain, the inflammatory site of the central nervous system, and cause damage to hippocampal cells, thereby causing cognitive impairment in mice. Isoflurane can cause a decrease in brain neurons, increase fiber A-B, and impair directionality and understanding. Studies have shown that Isofran can only cause memory loss, not retrograde memory loss. In rats under anesthetic concentration, long-term repeated inhalation of halothane, sevoflurane, and desflurane may cause changes in behavior. Among them, desflurane had the greatest impact on the learning and memory of mice. Inhalation anesthetic desflurane may change the appearance of specific proteins in the brain tissue cells of mice, part of which involves the transportation and metabolism of cysts. This change also occurred 7 hours after anesthesia. This is because inhaled anesthetics may affect the central nervous system. Neural function provides important molecular elements (iv). Long-term exposure to N : 0 will promote the death of rat nerve cells. This effect is related to the hindrance of NMDA receptor function.

#### 2.4.2. Intravenous Anesthetics

Propofol is widely used to introduce and maintain anesthesia, and it may occur after the patient's surgery. 100–150 mg/kg of propofol is often used for the introduction and maintenance of general anesthesia. 100–150 mg/kg preventive drugs may also cause retrograde memory loss, which can easily be forgotten within 3 hours. According to research, after propofol anesthesia in elderly patients, 9.4% of patients developed POCD within one week after surgery, and 7.8% of patients developed POCD within 3 months after surgery. Experimental studies have found that the application of preventive drugs in nerve cell culture can reduce GABAergic neurons, prolong the use time, and also kill GABAergic neurons and suggest that propofol does not promote the development of the nervous system. Many areas of the brain are involved in learning and memory, such as the joint areas of the cerebral cortex, hippocampus, and amygdala [33]. Male rats were randomly divided into two groups after destruction of the basal amygdala complex. The memory capacity of the prevention group was not significantly different from that of the prevention group, but the memory capacity of the preventive dysfunction group decreased, suggesting that the memory damage point caused by propofol may be the main complex of the amygdala.

## 3. Experiment on the Relationship between General Anesthetics and Postoperative Cognitive Dysfunction

### 3.1. Subject

We selected in our hospital 100 patients who planned to undergo elective gastrointestinal laparoscopic surgery under general anesthesia from March 2019 to November 2019. The operation time was more than 2 hours, and the age was ≥16 years. The ASA classification of patients was I-III.

Object exclusion criteria are the following:

1. People with a history of mental or neurological diseases, a history of long-term alcohol and drug abuse, and long-term use of opioids or stabilizers.
2. Patients with severe heart, lung, brain, liver, and kidney function abnormalities, as well as patients with history of diabetes, stroke, and so forth.
3. Small cog test confirming the existence of cognitive impairment and the examination score of patients with less than 20 points (due to China's national conditions, the age of the enrolled patients is generally older and their education level is lower, so 20 points is taken as the critical value).
4. Patients with deafness or blindness who are unable to complete the simple intelligence status scale.
5. Patients who refuse the test or cannot complete the scale test due to other reasons.
6. Patients who are allergic to the anesthetic drugs that need to be used during the experiment and have a family history of malignant high fever or a history of malignant high fever. The test subjects were included in strict accordance with the appeal criteria.

Regarding index testing standards, the detection basis is based on the BIS monitoring of the depth of anesthesia in the experimental group, the incidence of POCD on the 1st, 5th, 10th, 50th, and 200th days, discharge time and the incidence of POD on the 1st to 10th day after the operation, postoperative hospital stay, patient satisfaction, and other indicators.

### 3.2. Experimental Grouping

#### 3.2.1. Test Group

BIS was used to monitor the depth of anesthesia during the operation of the enrolled patients. The anesthesiologist maintained an anesthesia depth index of 40–60 during the whole process and obtained outcome indicators such as postoperative cognitive dysfunction and the incidence of postoperative delirium.

#### 3.2.2. Control Group

The BIS, which was blocked by a black curtain, was used to monitor the depth of anesthesia during the operation of the enrolled patients. The anesthesiologist was not aware of the changes in the value. During the whole anesthesia, the appropriate depth of anesthesia was maintained according to clinical experience and outcome indicators such as the incidence of postoperative delirium. The patients were divided into test group and control group. The two groups were divided into 50 patients by a randomized control plan. First, physician A designed the experimental grouping and experimental anesthesia plan and put it in an envelope. Second, physician B strictly followed the exclusion criteria to screen the test subjects and extract the corresponding experimental groupings and experimental protocol envelopes. Third, anesthesiologist C implemented the anesthesia program according to the envelope contents and recorded the experimental data. Fourth, physician D treated both groups of patients. Postoperative cognitive dysfunction and postoperative delirium and other outcome indicators were evaluated and recorded after the operation. Finally, physician E collected, sorted, counted, and analyzed all the data and obtained the test results. Among them, physicians A, B, C, D, and E all independently implemented the trial protocol and were unaware of other physicians' trials.

### 3.3. Statistical Analysis

This experiment uses SPSS 17.0 for statistical analysis. The measurement data is expressed by the average standard deviation (*x* ± *s*). *t*-test is used to compare the results of the two groups for statistical analysis. *p* < 0.05 is statistically significant. The measurement data is expressed as a ratio; and the two groups are compared with the chi-square test, and *p* < 0.05 is statistically significant.

## 4. Relationship between Artificial-Intelligence-Based General Anesthetics and Postoperative Cognitive Dysfunction

### 4.1. Relationship between Deep Anesthesia and Postoperative Cognitive Dysfunction

The comparison of the basic preoperative data of the two groups of patients is shown in Table 1 and Figure 1.

This trial is planned to enroll 100 patients, of which 2 patients in the BIS group withdrew from the trial because the anesthesia time was less than 2 hours, and, in the control group, 2 patients temporarily cancelled the operation, 2 patients were anesthetized for less than 2 hours, and 1 patient was deaf and withdrew from the trial. Finally, 48 patients were included in the BIS group and 45 patients were included in the control group. It can be seen from the above table that there is no significant difference in the basic conditions of the two groups of patients in age, gender, height, weight, BMI index, ASA classification, and educational level. However, there are significant differences in the history of surgical anesthesia between the two groups, which may be due to the fact that there are more patients in the control group who have undergone secondary gastrointestinal surgery, so the results of the two groups are different. However, at present, compared with the time of anesthesia, the more important effect on the cognitive dysfunction of patients after surgery may be the time of anesthesia. Secondly, it can be seen from the data of the appeal that this experiment included two groups of patients. The control variables in the overall comparison are relatively good; therefore, although the unified variables cannot be controlled perfectly, this study is still feasible and credible, and most of the current studies have not excluded patients with secondary operations or secondary anesthesia.

Statistics and calculations of postoperative results obtain postoperative POD and POCD, as shown in Tables 2 and 3 and Figure 2.

It can be seen from the above chart that the incidence of postoperative delirium in the two groups of patients was low, and the incidence of patients in the two groups was 0 on the 7th, 9th, and 10th days after the operation. In general, the two groups were compared. There is no significant statistical difference.

Finally, the patient's satisfaction with anesthesia during the hospitalization period was counted. The results are shown in Table 4 and Figure 3.

It can be seen from the above chart that there is no significant difference in the postoperative hospital stay between the two groups, but there is a significant difference in the degree of satisfaction with anesthesia between the two groups. Among them, the overall satisfaction of the BIS group is relatively high in 48 patients. 45 patients were satisfied, and only 6.25% were dissatisfied. However, in the control group, 40 of the 45 patients were satisfied with the anesthesia effect, and 11.11% were dissatisfied.

### 4.2. Relationship between the Recovery Period of General Anesthesia and POCD

Only use creatine sodium phosphate intravenous injection, lead patients to adjust their mood, control sodium intake, monitor weight, give Flomid diuretics for a long time, reduce the burden on the heart, and instruct patients to follow other treatments for left heart failure in the past instructions for treatment. According to the indicators of imaging and cardiac function and the patient's recovery, as a process of treatment, it is instructed to conduct periodic breathing and muscle relaxation training 2 to 3 times a day. According to the treatment of the comparison group, Qiliqiangxin capsules can strengthen the heart, treat diuresis, and dilate blood vessels by oral administration. This is the process of treatment, with 2∼3 capsules each time, 2∼3 times a day.

During hospitalization, clinical manifestations, average length of stay, and complication rate of the two groups are shown in Table 5, Figure 4, and Table 6.

For LVEF changes in the two groups during treatment, 20 cases in the treatment group were markedly effective, 18 cases were effective, and 2 cases were ineffective. In the control group, 12 cases were markedly effective, 18 cases were effective, and 10 cases were ineffective. 14 cases were markedly effective in cardiac function, 28 cases were effective in treatment, 24 cases were markedly effective in the control group, 8 cases were effective, and 3 cases were ineffective; for NBP changes, 30 cases were markedly effective in the treatment group and 12 cases were effective; 14 cases in the control group were effective, 18 cases were effective, and 8 cases were ineffective. According to clinical signs, left ventricular ejection fraction, and cardiac function, the total effective rate is calculated, as shown in Table 7 and Figure 5.

In this trial, the treatment group was treated with creatinine phosphate sodium, and the treatment group was combined with oral Qiliqiangxin capsules: the time until the clinical symptoms recovered, the average treatment time, and the incidence of complications were significantly shorter and always effective treatment is more important than the control group. The combination of Qiliqiangxin capsules and creatine sodium can improve the clinical effects of left heart failure in the elderly and help patients recover quickly.

## 5. Conclusions

At present, the incidence of postoperative cognitive dysfunction is increasing with the increase of the aging population. At present, scholars all over the world have conducted extensive research on this topic, and the correlation between the depth of anesthesia and postoperative cognitive dysfunction is currently studied less. There is still no clear pathogenesis or treatment for postoperative cognitive dysfunction. Starting from the depth of anesthesia, this experiment hopes to provide a new perspective for the treatment of POCD.

POCD is a general complication of anesthesia. There are other complications such as delayed recovery, long-term hospitalization, increase in medical expenses, and even an increase in postoperative mortality. Therefore, the prevention and treatment of POCD are very important, and clinicians must pay great attention to them. Because of the long cycle of neurodegenerative diseases, clinical research is almost retrospective, so more samples are needed. Among many factors affecting POCD, multifocus clinical studies have shown that the etiology of POCD cannot be ignored in general anesthetics. Facing the occurrence of POCD, anesthesiologists should take reasonable medication according to the actual situation.

In experimental studies, we found that general anesthesia has a special effect on postoperative cognitive function. However, any research method has certain limitations, and changes in the environment will also cause some differences in results. For example, when a simple intelligence test is used to check the cognitive function changes of elderly patients after surgery, if the patient does not cooperate, it will affect the experimental results: in the process of animal experiments, sometimes the temperature and intensity of ambient light will also cause large experimental results. Not the same. Therefore, we must design scientific experiments, carefully and accurately observe the experimental process, objectively analyze the experimental results, and draw reasonable conclusions based on clinical practice.

## Figures and Tables

**Figure 1:** Comparison of preoperative data between the two groups.

**Figure 2:** Basic situation of POCD patients.

**Figure 3:** Comparison of satisfaction with anesthesia.

**Figure 4:** Comparison of clinical manifestations and length of stay in the two groups.

**Figure 5:** Comparison of total effective rates between the two groups.

**Table 1:** Comparison of preoperative data between the two groups.

	BIS Group	Control group	*t*/*x*2	*p*
Age	55 ± 15	53 ± 11	0.9	0.372
Height	165 ± 8	162 ± 6	1.6	0.110
Body weight	56 ± 10	57 ± 13	0.9	0.38
Culture	7 ± 3	6 ± 4	1.0	0.33
BMI	22 ± 4	21 ± 3	0.5	0.64
Male	28	20	—	—
Female	20	25	—	—
ASI Class I	9	7	—	—
ASI Class II	21	27	—	—
ASI Class III	8	2	—	—
Have a history of anesthesia	20	29	—	—
No history of anesthesia	28	16	—	—

**Table 2:** Situation of POD patients.

Project	BIS Group (%)	Control group (%)	*x*2	*p*
Day 1	14.3	6.5	0.46	0.520
Day 2	6.8	4.3	0.22	0.490
Day 3	4.3	0	—	0.331
Day 4	3.3	0	—	—
Day 5	2.4	0	—	—
Day 6	1.2	0	—	1
Day 7	0	0	—	—
Day 8	1.2	0	—	1
Day 9	0	0	—	—
Day 10	0	0	—	—

**Table 3:** POCD situation.

Project	BIS Group (%)	Control group (%)	*x*2	*p*
Day 1	22.4	13.4	0.933	0.343
Day 5	5.3	17.3	1.662	0.197
Day 10	7.9	8.8	0.000	1
Day 50	8.2	23.1	3.210	0.067
Day 200	7.9	28.7	4.983	0.023*∗*

^*∗*^ *p* < 0.05, which is statistically significant.

**Table 4:** Comparison of satisfaction with anesthesia.

Satisfaction level	BIS Group	Control group
Very satisfied	12	10
Quite satisfied	23	15
Satisfied	10	15
Not satisfied	3	5

**Table 5:** Comparison of clinical manifestations and length of stay in the two groups.

Grouping	Therapy group	Control group
Difficulty breathing	3 ± 1.2	6 ± 1.2
Tired	5 ± 1.3	10 ± 1.2
Anxiety	4 ± 1.3	9 ± 1.4
Average length of stay	8 ± 1.1	12 ± 1.6

**Table 6:** Comparison of complications.

	Therapy group	Control group	*p*
Complication (*n*)	2	5	<0.05
Complication rate (%)	3.3%	14.6%	<0.05

**Table 7:** Comparison of total effective rates between the two groups.

Grouping	Therapy group	Control group
N	40	40
Markedly effective	20	12
Effective	18	18
Invalid	2	10
Total effective rate (%)	95	75

## Data Availability

No data were used to support this study.
